RETRACTED

# Influence of MRI on Diagnostic Efficacy and Satisfaction of Patients with Alzheimer's Disease

**DOI:** 10.1155/2021/9038784

**Published:** 2021-11-08

**Authors:** Zheng Dong, Xinyu Yang, Liming Chang, Xin Song, Xiangchun Li, Jiantao Wang, Juntao Li

**Affiliations:** Department of Radiology, Tangshan Gongren Hospital, Tangshan, Hebei 063000, China

## Abstract

**Objective:**

To inquire into the influence of magnetic resonance imaging (MRI) on the diagnostic efficacy and satisfaction of patients with Alzheimer's disease (AD).

**Methods:**

This study included 42 healthy people (control group) and 66 patients with AD (AD group). The hippocampus volume, temporal sulcus spacing, left-right brain diameter, brain lobe volume, hippocampal height, temporal horn width, lateral fissure width, and degree of leukoaraiosis were all measured using an MRI scan. After diagnosis, the satisfaction of patients in both arms was investigated and the satisfaction degree was recorded.

**Results:**

Compared with the control group, the left and right hippocampal volumes and hippocampal height of AD patients were smaller, while the temporal sulcus spacing, temporal horn width, lateral fissure width, and left-right brain diameter were remarkably higher. A statistical difference was present in the degree of leukoaraiosis between the two arms. The frontal and temporal lobe volumes of AD patients were notably lower while the volumes of parietal and occipital lobes were similar, versus the control group. The total satisfaction was 83.33% in the control group and 86.36% in the AD group, with no statistical difference between the two arms.

**Conclusions:**

MRI can effectively mine the brain information of AD patients with a high patient satisfaction, which has potential value in clinical application.

## 1. Introduction

Alzheimer's disease (AD) is a common neurodegenerative disease characterized by neurite plaques and neurofibrillary tangles (NFT) that cause amyloid peptide accumulation in the brain, which significantly reduces an individual's ability to think and perform independent daily activities [1]. A meta-analysis [2] indicates that the prevalence rate of AD in Europe is 5.05%, with an annual incidence of 11.08 cases per thousand. The statistical prevalence of AD from 1994 to 2012 was 14.6-14.7%, while the annual incidence was 2.2-2.8% [3]. According to a cross-sectional study [4], the prevalence of AD in China is about 4%, which is strongly related to gender, age, education level, and region. Besides, it is shown that AD is obviously correlated with age. A study [5] predicts that increased life expectancy in society will lead to a high prevalence of AD in the future. The majority of instances of Alzheimer's disease are caused by hereditary factors, although cerebrovascular disorders, diabetes, hypertension, and dyslipidemia all enhance the chance of developing the illness [6].

RETRACTED

The current clinical diagnosis of Alzheimer's disease relies on signs, symptoms, blood markers, pathology, and imaging data to make the determination. One of them is magnetic resonance imaging (MRI), a noninvasive technique that may give a wealth of information on the brain in many dimensions, including architecture, function, and metabolism. Alzheimer's disease (AD) is anticipated to become routinely evaluated by MRI-based brain atrophy diagnosis [7]. Diagnostic accuracy for Alzheimer's disease may be greatly improved by using magnetic resonance imaging (MRI) to look for pathological characteristics and biomarker levels. This information can then be used to guide the development of new treatments. One study [8] suggested that the MRI-based deep learning method was 99.10 percent accurate, 99.80 percent sensitive, and 98.40 percent specific in distinguishing AD from healthy individuals. Another study [9] assessed the accuracy of multimodal MRI in diagnosing AD at 98.58%.

The diagnostic treatment of Alzheimer's disease by MRI is still in the early stages of development. There were 66 Alzheimer's sufferers and 42 healthy individuals in this study. Combined with MRI, the brain images of the two arms were scanned and the differences were compared, in order to highlight the significant efficacy of MRI in distinguishing AD patients from controls and to analyze its impact on the diagnostic satisfaction of patients, so as to provide reliable scientific research data for MRI diagnosis of AD.

## 2. Materials and Methods

### 2.1. General Information of Participants

This study included 66 AD patients (AD group) and 42 healthy controls (control group). The control group had 23 males and 19 females, with an average age of 70.12 ± 5.10 years and an average course of disease of 2.26 ± 0.60 years; as far as their educational degree was concerned, there were 25 cases of junior middle school or below, 12 cases of technical secondary school or senior high school, and 5 cases of junior college or above. In the AD group, the male to female ratio was 37 : 29, the mean age was 70.21 ± 4.32 years, and the average course of disease was 2.23 ± 0.59 years. As a result, there were 39 students in junior middle school or below, 16 in technical secondary school or senior high school, and 11 in junior college or above who were affected. When examining a variety of factors including age and education level and a patient's body mass index (BMI), the researchers found that the two groups were quite comparable. This suggests that more research might be done to compare the results (Table 1). The inclusion criteria for Alzheimer's disease patients were age more than 60, the ability to conduct an MRI examination with the assistance of family members or medical professionals, the absence of a history of brain surgery, and complete clinical data. Patients with Alzheimer's disease are not eligible if they have any of the following conditions: congenital dementia, craniocerebral dysplasia, drug-induced dementia, mixed dementia, and MRI contraindications due to intraorbital foreign bodies, cerebral artery clamps, or metal joint implantation after craniocerebral surgery.

RETRACTED

### 2.2. Inspection Methods

Both groups received MRI examination. After verifying that there were no MRI contraindications, the patient was helped into a supine posture with his or her hands on his or her sides and head advanced. An MRI scanner with a 16-channel orthogonal head coil was used to image the brain. To keep the cross-sectional positioning cursor in line with both eyes, the subject's head was put in a head coil. Sagittal cursor was positioned in the midsagittal plane of the head, and sponge pads were put on both sides of the posterior head for appropriate fixing during examinations.

### 2.3. Outcome Measures

1. The difference of hippocampal volume was compared between the AD group and the control group. The margin of hippocampus was determined layer by layer, and its area was calculated. The volume of hippocampus was equal to the sum of the areas of each layer ∗ layer thickness
2. The differences of temporal sulcus spacing and left-right brain diameter were observed and recorded
3. The degree of leukoaraiosis (grades 0-4) detected by parallel diffusion tensor imaging scan was compared. Grade 0: no leukoaraiosis lesions, grade 1: 1-2 lesions, grade 2: 3-5 lesions, grade 3: >5 lesions, and grade 4: fusion lesions
4. The volume differences of frontal, temporal, parietal, and occipital lobes were analyzed by MRI coronal scanning. The frontal, temporal, parietal, and occipital lobes' boundaries were determined layer by layer to calculate their area. Brain lobe volume = sum of the areas of each layer∗layer thickness, and the volume of each lobe was expressed as the proportion of it to the cranial cavity volume
5. Linear measurements of hippocampal height, temporal horn width, and lateral fissure width were taken and compared. On oblique coronal SE T1WI, the height of the hippocampus was the maximum vertical diameter of bilateral hippocampi, the width of temporal horn was the maximum width of lateral ventricle temporal horn, and the width of lateral fissure was the greatest width of bilateral lateral fissure cisterna
6. All the participants were investigated for satisfaction, and the evaluation was divided into very satisfied, satisfied, and dissatisfied, with total satisfaction = (very satisfied + satisfied) cases/total cases in each group

RETRACTED

### 2.4. Statistical Analysis

This research used the SPSS statistical software to examine participant picture data. Meanvariance and number of instances were used to convey quantitative information. The independent sample *t* test (two-tailed test) was used to examine the statistical differences in measuring data across the groups, and the Chi-square test was used to compare the counting data. The 95% confidence interval was used, and a *p* value of less than 0.05 indicates a significant difference.

## 3. Results

### 3.1. Comparison of MRI-Based Measurement of Hippocampal Volume

In Figure 1, MRI brain pictures of patients are shown. When compared to controls, AD patients had significant hippocampal atrophy. The MRI-based assessment of hippocampus volume was compared in this research. As shown in Table 2, the left and right hippocampal volumes of the AD group were 1.99 ± 0.11 cm^3^ and 1.92 ± 0.14 cm^3^, respectively, significantly lower than those of the control group (2.61 ± 0.08 cm^3^ and 2.68 ± 0.12 cm^3^).

### 3.2. Comparison of MRI-Based Measurement of Temporal Sulcus Spacing and Left-Right Brain Diameter

MRI-based measurement of temporal sulcus spacing and left-right diameter of brain were compared. The results (Table 3) identified that the temporal sulcus spacing and left-right brain diameter in the control group were 23.11 ± 4.77 mm and 116.56 ± 10.42 mm, respectively, significantly lower than those in AD patients (31.07 ± 4.57 mm, 124.82 ± 16.52 mm; *p* < 0.05).

### 3.3. Comparison of MRI-Based Measurement of Leukoaraiosis Degree

In this study, the leukoaraiosis degree obtained from MRI images was compared between the two arms. The results (Table 4) revealed 34 cases of grade 0 and 7 cases of grade 1 in the control group, while in the AD group, the number of cases with grades 0, 1, 2, 3, and 4 was 25, 28, 4, 6, and 3, respectively. The degree of leukoaraiosis between the two groups was markedly different (*p* < 0.001).

### 3.4. Comparison of MRI-Based Measurement of Cerebral Lobe Volume Ratio

In this study, MRI was used to obtain the volume ratio of each lobe of two groups, and the results are shown in Table 5. The volumes of frontal, temporal, parietal, and occipital lobes in AD patients were 12.81 ± 1.62%, 3.13 ± 2.04%, 8.49 ± 1.72%, and 4.57 ± 2.06%, respectively, while those in the control group were 16.44 ± 2.81%, 5.31 ± 1.31%, 8.09 ± 1.59%, and 4.26 ± 0.99%, respectively. Frontal and temporal lobe volumes were evidently lower in AD patients than in controls (*p* < 0.001), but the volumes of parietal and occipital lobes differed insignificantly (*p* > 0.05).

RETRACTED

### 3.5. Comparison of MRI-Based Measurement of Hippocampus Height, Temporal Horn Width, and Lateral Fissure Width

Hippocampus height, temporal horn width, and lateral fissure width were measured using MRI in this research. The results (Table 6) identified noticeably lower hippocampal height while remarkably higher width of temporal horn and lateral fissure in AD patients than in controls (all *p* < 0.001).

### 3.6. Influence of MRI on Satisfaction of AD Patients

Also, this study conducted a satisfaction survey for the enrolled participants (Table 7). With a total satisfaction rating of 83.33 percent in the control group, 25 patients were extremely pleased, 10 cases were moderately satisfied, and 7 cases were dissatisfied. With a total satisfaction rating of 86.36 percent in the AD group, 38 patients were extremely pleased, 19 instances were moderately content, and 9 cases were dissatisfied. It identified no statistical difference in satisfaction between the two arms (*p* = 0.666), indicating that AD patients had no obvious rejection of MRI diagnosis.

## 4. Discussion

AD is a significant financial burden on the world economy, and there are no specific therapeutic options [10]. Alzheimer's disease (AD) will likely become more common in the next decades. As a result, useful biomarkers for early illness detection should be investigated [11]. Although computed tomography (CT) can assess tissue structure linearly and image brain atrophy, its soft tissue resolution is restricted. Because of advancements in MRI technology, it becomes much easier to map the brain's intrinsic network structure. Because MRI can clearly show the anatomical structure of the brain and provide three-dimensional information on the patient's brain tissue, it has become one of the most popular studies in the medical field. MRI methods, especially functional magnetic resonance imaging, are a noninvasive diagnostic tool that does not need the use of contrast agents or exposure to radiation, making them repeatable in longitudinal investigations [12]. At present, MRI still needs a lot of routine clinical applications to prove its diagnostic value in AD.

Hippocampal atrophy is a clinicopathological feature that distinguishes AD from other vascular dementia diseases. An *in vivo* longitudinal MRI study [13] demonstrates a significant reduction in basal forebrain volume in patients with AD. This study analyzed MRI-based measurement of hippocampus alterations. Compared with the control group, the height of hippocampus and the volume of left and right hippocampus of AD patients shrank notably, as well as the volume of frontal and temporal lobes. Using structural MRI, Pennanen et al. [14] discovered substantial hippocampal shrinkage in AD patients. Patients with Alzheimer's disease have substantial grey matter loss in the hippocampus. AD patients were shown to have significant leukoaraiosis in this research, which may be linked to hippocampus atrophy [15]. There was considerable variability in white matter distribution, which was significantly associated with illness types and lesion degrees, according to a clinical research using advanced diffusion MRI. For in vivo white matter imaging, magnetic resonance imaging (MRI) is ideal. Alzheimer's disease (AD) is characterized by a widening of the left-right brain diameter, widening of the temporal horn, and widening of the lateral fissure in the temporal lobe, all of which may be caused by amyloid buildup in the brain, further accelerating the disease. These differences indicate the great potential of MRI in excavating neurodegenerative areas. Because there was no significant difference in diagnostic satisfaction between the two groups, MRI offered a lot of promise for increasing patient compliance because there was no apparent rejection.

RETRACTED

Although this study conducted a diagnostic analysis of AD based on MRI, there are still some limitations. At present, MRI still faces great economic and time costs and is influenced by environmental factors. A study [16] suggests that convolutional neural network combined with MRI technology can accelerate the routine application of MRI in early AD diagnosis. Hence, we will further discuss the clinical application cost of MRI in combination with other diagnostic modalities in the future. In addition to the information of hippocampus and cerebral lobes involved in this study, patients' cerebral hemodynamic parameters may also be obtained using MRI. According to Basaia et al. [17], arterial spin labelling MRI may be useful in understanding the aetiology and early detection of Alzheimer's disease by monitoring cerebral blood flow. Additionally, understanding changes in MRI-based measurements of cerebral hemodynamic parameters will aid in the differentiation of Alzheimer's disease from mild cognitive impairment [18]. This is also an area on which the authors want to do more study in the future. As a result of the study's sample size limitations, we want to recruit additional participants in future research in order to provide more accurate scientific data. All in all, this paper demonstrates that MRI can provide a wealth of imaging and data information for clinical diagnosis and risk stratification by deeply mining the brain information of AD patients. MRI-based diagnostic strategy can effectively distinguish patients' hippocampal atrophy, temporal horn width, lateral fissure width, temporal sulcus spacing, left-right cerebral diameter, and leukoaraiosis degree. Moreover, patients' high satisfaction with MRI diagnosis will effectively promote patient compliance. Therefore, MRI diagnosis of AD is of high clinical application value.

RETRACTED

## Figures and Tables

**Figure 1:** MRI images of patients with Alzheimer's disease. Temporal horn width was measured on transverse T1WI, T2WI, and FLAIR images, and hippocampus height was measured on oblique coronal T2WI images.

**Table 1:** General information.

	Control group	AD group	*χ* ^2^/*t*	*p*
*n*	42	66		
Gender			0.02	0.895
Male	23	37		
Female	19	29		
Age/year	70.12 ± 5.10	70.21 ± 4.32	0.102	0.919
Course of disease/year	2.26 ± 0.60	2.23 ± 0.59	0.263	0.793
Education level			0.579	0.749
Junior high school and below	25	39		
Technical secondary school and high school	12	16		
Junior college or above	5	11		
BMI/kg·m^2^	20.28 ± 0.66	20.29 ± 0.53	0.105	0.917
History of smoking			0.327	0.568
Yes	18	32		
No	24	34		
History of alcoholism			0.05	0.820
Yes	15	25		
No	27	41		

**Table 2:** Comparison of hippocampal volume between two groups.

	Control group	AD group	*t*	*p*
*n*	42	66		
Left hippocampus/cm^3^	2.61 ± 0.08	1.99 ± 0.11	30.61	<0.001
Right hippocampus/cm^3^	2.68 ± 0.12	1.92 ± 0.14	29.84	<0.001

**Table 3:** Comparison of temporal sulcus spacing and left-right brain diameter between two groups.

	Control group	AD group	*t*	*p*
*n*	42	66		
Temporal sulcus spacing/mm	23.11 ± 4.77	31.07 ± 4.57	8.611	<0.001
Left-right brain diameter/mm	116.56 ± 10.42	124.82 ± 16.52	2.893	0.005

**Table 4:** Comparison of the degree of leukoaraiosis between two groups.

	Control group	AD group	*χ* ^2^	*p*
*n*	42	66	22.35	<0.001
Grade 0	34	25		
Grade 1	7	28		
Grade 2	0	4		
Grade 3	0	6		
Grade 4	0	3		

**Table 5:** Comparison of brain lobe volumes between two groups.

	Control group	AD group	*t*	*p*
*n*	42	66		
Frontal lobe (%)	16.44 ± 2.81	12.81 ± 1.62	8.540	<0.001
Temporal lobe (%)	5.31 ± 1.31	3.13 ± 2.04	9.764	<0.001
Parietal lobe (%)	8.09 ± 1.59	8.49 ± 1.72	1.528	0.129
Occipital lobe (%)	4.26 ± 0.99	4.57 ± 2.06	1.620	0.108

**Table 6:** Comparison of hippocampal height, temporal horn width, and lateral fissure width between two groups.

	Control group	AD group	*t*	*p*
*n*	42	66		
Height of hippocampus	16.36	10.65	11.93	<0.001
Width of temporal horn	3.57	5.06	8.316	<0.001
Width of lateral fissure	4.37	5.23	4.463	<0.001

**Table 7:** Comparison of satisfaction between two groups.

	Control group	AD group	*χ* ^2^	*p*
*n*	42	66		
Very satisfied	25	38		
Relatively satisfied	10	19		
Dissatisfied	7	9		
Overall satisfaction	35 (83.33)	57 (86.36)	0.187	0.666

RETRACTED

## Data Availability

The data used to support the findings of this study are included within the article.
